# Evidence-based nursing practice and improving pediatric patient care outcomes in the prevention of infection transmission: Emergency department findings

**DOI:** 10.1371/journal.pone.0305001

**Published:** 2024-06-21

**Authors:** Omar Mohammad Ali Khraisat, Ahmad M. Al-Bashaireh

**Affiliations:** 1 Faculty of Nursing, Al-Ahliyya Amman University, Amman, Jordan; 2 Faculty of Health Sciences, Higher College of Technology, Abu Dhabi, United Arab Emirates; Mutah University, JORDAN

## Abstract

**Background:**

Reducing the risk of infection transmission by getting emergency care for pediatric patients is a challenging task.

**Aim:**

The study aim was to assess emergency nurses’ readiness to provide care for pediatric patients with infectious diseases.

**Method:**

Two hundred Jordanian emergency department nurses were surveyed using a descriptive design.

**Results:**

The study revealed that insufficient safety and infection control procedures were put into place, starting with family support to allow nurses to work 145 (78%), family care plans intended to assist caregivers 139 (74.7%), the availability of respiratory protection and a backup plan for standard precautions, training requirements, and equipment 131 (70.4%), create a unit pandemic safety strategy 124 (66.7%), have a plan for emergencies for at-risk staff 116 (62.4%), have a hospital pandemic safety plan 113 (60.8%), manage inventory 102 (54.8%), use reuse guidelines if there will be severe shortages 99 (53.2%), create a strategy for nurses’ access to healthcare for themselves and their families 96 (51.6%), and end with any required system updates for new policies 88 (47.3%). Staff nurses made up a large proportion of participants (145; 78%; 115; 62.8%) who said they lacked experience with care for pediatric patients with infectious illnesses who were critically sick. A 62.8% of nurses reported they did not have training in infectious disease emergency prevention and control for pediatric patients. What nurses prioritize it was determined that the concept of crisis standards of care (34.9%) was the most important educational topic for training emergency room nurses to care for pediatric patients who are critically ill with infectious infections, while the clarity of communication pathways was ranked lowest.

**Conclusion:**

More training and support are needed for emergency room nurses to properly care for children’s patients with infectious illnesses.

## Introduction

An essential component of evidence-based nursing practice is enhancing the outcomes for pediatric patients in terms of infection transmission prevention [1]. One of the biggest challenges in emergency care is still infection prevention [2]. Patients range in acuity from the otherwise healthy to the seriously ill, presenting with nonspecific diseases, mainly in children. Compared to adults, children are much more likely to present to the ED with non-specific fever [2]. They must be visually checked upon arrival by a competent staff member, which should not delay care and create a crowded line [3]. Children who are really ill are more likely to come by car than by ambulance than adults.

Pediatric populations are especially vulnerable to the spread of infections because: children’s immune systems are still developing and may not be as strong as adults’; they have a higher transmission rate; some infectious diseases can have long-term health effects on children; and children can act as reservoirs for infectious diseases, passing them on to older people or people with underlying medical conditions [3,4].

Healthcare professionals must examine a child’s ears and throat up close, unlike when examining an adult. Compared to adults, children undergo examinations significantly more frequently, and this, together with crying (especially during evaluation), may accelerate the spread of infections [2]. In particular, when younger children are more tactile, tend to wander more, and may not accept masks. Cohorting in waiting rooms while experiencing social distance is so challenging [3]. Because of their responsibilities to the upbringing of other children, professionals may be caring for more sick people. Toys and other objects are commonly utilized as distractions in waiting spaces, which raises the infection rate [2].

Infectious illness emergencies, especially those that reach epidemic levels, are influenced by the biological agent’s features, the extent of exposure, the transmission method, and intentionality [1,4]. The moment the patient was admitted, these infections are neither present nor incubating [3]. Nurses faced with severe time and resource constraints, medical decision-making and risk assessment are frequently dependent on scarce and changing facts. Closely spaced from one another, patients await diagnosis, treatment, and disposition [2]. Healthcare-associated infections increase patients’ mental distress and functional incapacity and, in some situations, can result in life-limiting illnesses [2,3]. According to the World Health Organization (WHO), 4% to 10% of patients who are admitted to a hospital will get a nosocomial infection [5].

Pandemics, epidemics, and outbreaks of transmissible illnesses are examples of emergencies [5]. Effective response plans for all infectious diseases, including those that become pandemics, must be created by the facility [6]. Emergency departments must limit visitor access to ensure safe social distance [4]. For persons who are seriously ill, near death, are deemed socially vulnerable, or are minors who will require at least one competent adult, exception may be taken into account on an individual basis [4]. Additionally, nurses should consider infection prevention strategies since patients should not experience a fear as a result of using Personal Protective Equipment (PPE) [4].

For pediatric patients and other frail individuals, this is essential. It is recommended to employ a variety of forms (posters, information booklets, etc.) to clearly convey PPE [4]. At all PPE levels, nurses should be immediately recognized by their name and position [7,8]. Since nurses spend the most time with pediatric patients, they are the foundation of the emergency care team and are in charge of providing high standards of care. The scale of exposure, reach, and effectiveness of nurses’ contributions to the delivery of emergency services for infectious diseases has been particularly important [7–9]. Innovative and efficient care strategies for infectious disease emergencies have long been pioneered by nurses [10].

It is significant to remember that evidence-based nursing practice in infection prevention is a developing field, and these findings are not all-inclusive [5]. To give pediatric patients the best care possible and enhance their outcomes while limiting the spread of infections in the emergency room, nurses should keep up to date on the most recent findings and recommendations [11,12]. Nurses should be informed of isolation precaution guidelines and ensure that they are followed, including hand hygiene procedures and PPE use, to lower the risk of infection transmission [3]. It is essential that nurses supervise and ensure compliance with environmental cleaning procedures in a proactive manner. Infection prevention methods also need to incorporate patient and family education initiatives and open channels of communication between healthcare providers [3].

Besides, nurses receive ongoing instruction in infection control methods, including hand washing, appropriate use of personal protective equipment (PPE), and isolation measures, through education and training that evaluates their needs [4]. Educate patients and their families about the importance of vaccinations and additional infection control measures, including respiratory hygiene. Install surveillance and infection monitoring systems for medical infections [6]. Regularly analyzing and reporting infection rate data, identifying problem regions, and implementing preventative measures may halt the spread of illnesses [3,6].

Although, in pediatric care settings, nurses can successfully lower the risk of infections and enhance patient care outcomes by employing evidence-based practices [5]. As part of these evidence-based treatments, pediatric patients undergo a thorough assessment to determine the variables that make them more vulnerable to infections [1]. This could entail assessing their exposure risks, immunization status, underlying medical issues, and medical history [2]. Also, implementing infection prevention bundles, such as those that prevent surgical site infections (SSI), ventilator-associated pneumonia (VAP), and central line-associated bloodstream infections (CLABSI), improves children’s overall health [3].

Likewise, continuous quality improvement initiatives are used to monitor infection rates, pinpoint areas for improvement, and apply evidence-based treatments [4]. This may involve obtaining, evaluating, and offering feedback on data in order to enhance outcomes and encourage practice improvements [6]. By implementing these evidence-based approaches into nursing practice, infections in pediatric patients can be effectively prevented and controlled. This will improve the children’s entire health-care experience.

Further, the COVID-19 pandemic prompted nations to call on the medical community to prepare for emergencies and take preventative measures against infectious diseases [11]. Jordan stepped up its COVID-19 response in 2019, according to the Jordanian National Center for Epidemiology and Communicable Diseases Control (JCDC). Preventative interventions and emergency nursing care preparedness for pediatric patients in the event of an infectious disease emergency, however, are little understood [11].

In light of this, several areas still need to be evaluated and strengthened to support the growing readiness for epidemics and pandemics in the future. These include pediatric-specific research, the need for nurses to receive specialized training in pediatric epidemic and pandemic preparedness, the importance of effective stakeholder collaboration and communication for pediatric epidemic and pandemic preparedness, and the necessity of strengthening health information systems to gather, analyze, and share data on pediatric patients during pandemics.[11,12]. As well as, the issue with the state of evidence-based practice (EBP) in Jordan is that its application is restricted to a few initiatives in clinical practice and a few attempts to disseminate it through educational lectures, seminars, and journal clubs. No policy has been put in place to organize the integration of newly approved clinical related evidence that advances and improves the quality of care [13].

Thus, it is crucial to remember that the precise conclusions and approaches may change based on the environment, available resources, and infectious diseases that are common in a given area or emergency room. Therefore, enhancing pediatric patient outcomes in infection prevention within the emergency department requires maintaining current evidence-based guidelines and customizing interventions to the local environment. The purpose of this study was to assess the nurses’ readiness to provide care for pediatric patients with infectious diseases as well as their training requirements in such situations.

## Methods

### Study design and setting

Nursing emergency rooms’ readiness for caring for sick pediatric patients was assessed using a descriptive cross-sectional methodology in Jordan’s tertiary hospitals. In Jordan’s tertiary hospitals, pediatric patients can receive a range of emergency services in the country’s capital, Amman. These hospitals have dedicated pediatric sections and staff members who have experience providing care for children. In addition, Amman has a large number of tertiary hospitals that provide emergency care to over 4 million people, or 36% of Jordan’s population. Conveniently, nurses from the private and two governmental hospitals in Amman, Jordan’s capital, were chosen to participate in the study.

### Inclusion and exclusion criteria

Nurses who were not providing pediatric care, had previously taken part in a study similar to this one or had contact with the intervention under investigation, or who might have safety concerns or contraindications related to the study were excluded. All nurses who were providing pediatric care in Jordanian emergency departments (EDs) and could effectively communicate in the language(s) required for the study were eligible to participate.

### Sample

The research was carried out at the emergency rooms of three tertiary hospitals in Amman the capital of Jordan between February 2022 and August 2022. According to Cohen’s [14], a 200 participants was required for convenience sample based on power = 0.80, alpha = 0.05, and medium effect size = 0.25. The response rate is 93% (186 participants).

### Instrument

Self-reported anonymous questionnaires were used in the study. The questionnaire is divided into two parts. The first part of the questionnaire asks about age, gender, education level, years of experience, professional title, and whether or not the participant has received any formal training in infectious disease emergencies, specifically for pediatric patients who are severely ill with communicable diseases. Formal training refers to structured educational courses designed to equip participants with the knowledge, skills, and competencies needed to handle outbreaks, epidemics, and other infectious disease-related public health emergencies are referred to as formal training in infectious disease emergencies [6].

The Communicable Disease Pandemic Preparation Questionnaire (CDPPQ) for the infection prevention and control scale is included in the second part and was developed by the USA Health Care Coalition in 2019 [15]. The questionnaire has a total of 14 questions about the circumstances of infection prevention and control. Methods scale the responses with 1 indicating completion, 2 work in progress, and 3 work not yet begun. Additionally, component three was created by researchers and includes a ranking of the pandemic educational demands according to importance.

### Pilot study

To evaluate the instrument’s psychometric properties, a pilot study was conducted to determine how long the questionnaire would take to complete and how clear it would be. Within five to fifteen minutes, twenty nurses answered the questionnaire. The results of the pilot study were not included in the study. The alpha coefficient for the CDPPQ infection prevention and control scale reliability was 0.89. Cronbach alpha coefficient was 0.88, according to study by Al Haliq et al. (2022) [6]. The content validity of the questionnaire was assessed by two academic staff members who hold PhDs in pediatric health nursing.

### Data collection

After ethical permission was obtained from Al-Ahliyya Amman University (AAU). Following approval from the hospitals where the study was carried out, participants were contacted in private hospital rooms. All study participants who provided written consent got thorough information about the risks and benefits of the study. The survey in English was given out at the end of the shift. The study’s goals were explained to the participants. The questionnaire and a cover letter were given to them.

### Ethical considerations

The Al-Ahliyya Amman University’s Faculty of Nursing’s Scientific Research and Ethical Committee gave its ethical permission (D12/12/2021, MM 5). All study participants who provided written consent got thorough information about the risks and benefits of the study. It was assured to them that there was no risk. Also, individuals received guarantees that their participation in the study was entirely voluntary and that they could withdraw at any time without facing any consequences. The participants’ questionnaires were given numbers, kept in a locked location, and the data was entirely deleted once the study was over, providing those with further assurance that all the information gathered would remain anonymous. Completing and returning the questionnaire at the end of the shift implied the participant’s consent to participate in the study.

### Data analysis

Data were assessed using version 22 of SPSS [16] (Statistical Package for Social Science). Outliers, missing data, and entry errors in the data were scanned. Using descriptive statistics like frequency, percentage, mean, and standard deviation the sample’s characteristics were presented. There were no missing values or outliers.

## Results

A total of 200 questionnaires were surveyed, and 186 (93%) of them were returned. The majority of participants’ average age was 26.8 (SD: 3.4). Participants were mostly female (126; 67.7%), and 127; 68.3% held bachelor’s degrees. Additionally, 108 (58%) had more than five years of professional experience working in emergency departments. The majority of participants who work as staff nurses (145; 78%) reported they did not have training in infectious disease emergency prevention and control (115; 62.8%), indicating that education is necessary to care for pediatric patients in emergency rooms who are critically ill and have communicable diseases (Table 1).

**Table 1:** Demographic characteristics of participants’ (N = 186).

Variables	Frequency	Percentage
Age Mean (SD) 26.8 (3.4)		
Gender		
Male	60	32.3
Female	126	67.7
Educational degree		
Diploma degree	59	31.7
Bachelor’s degree	127	68.3
Professional experience in ED		
Less than 2 years	34	18.3
2–5 years	44	23.7
More than 5 years old	108	58
Professional title		
Charge nurse	41	22
Staff Nurse	145	78
Receive training in infectious disease emergency preventative procedures and control Yes No	71 115	38.2 62.8

### Emergency nursing readiness toward infectious diseases among pediatric patients

According to nurses, the greatest percentages of improperly implemented infection control measures were respectively included: “evaluate the need for family support to enable nurses to work (e.g., childcare)” 145 (78%),”provide specifics for family care plans that are intended to help caregivers by instructing them on how to supply the crucial information concerning childcare, school, medical care, and family activities” 139 (74.7%),”create a backup plan (Plan- B) that includes standard precautions, training requirements, and equipment” 131 (70.4%),”create a unit pandemic safety strategy and designate a safety officer to make any necessary modifications 124 (66.7%),”have a strategy for emergencies that includes job requirements and potential substitute responsibilities and locations for at-risk staff (such as pregnant employees and other designated risk categories) 116 (62.4%),”create a hospital pandemic safety plan, and designate a safety officer to make any necessary modifications113 (60.8%),”the medical supply members to be on the lookout for supply shortages 102 (54.8%),”create guidelines for the prudent use of N95 respirators/powered air-purifying respirators (PAPR) if severe shortages are coming up 99 (53.2%),”urging ED to make necessary arrangements for nurses’ access to medical care for themselves and their families 96 (51.6%),”teach personnel about infection management, and update regulations as needed 88 (47.3%) (Table 2).

**Table 2:** Emergency nursing readiness for pediatric patients with infectious diseases (N = 186).

Variable	Work in completed		Work in progress		Work not yet begun	
	Frequency	Percentage	Frequency	Percentage	Frequency	Percentage
Encourage all nurses to undergo N95 respirator fit testing.	52	28	68	36.6	66	35.5
Keep an eye on the availability of powered air-purifying respirators (PAPR), N95 respirators, and other infection control equipment.	41	22	98	52.7	47	25.3
Create a process for reporting both illness and absenteeism using the SBAR (Situation, Background, Assessment, Recommendation) documentation style. Establish guidelines for staff monitoring for indicators of illness (including self-reporting, self-quarantine, and start/end of shift evaluation).	59	31.7	79	42.5	48	25.8
Create a nurse return-to-work policy for those who become ill	41	22	75	40.3	70	37.6
Informing personnel about infection control and updating procedures as necessary	33	17.7	65	34.9	88	47.3
If adequate levels of respiratory protection are not available, create an emergency plan (e.g., standard precautions, training requirements, and equipment) (Plan- B).	20	10.8	35	18.8	131	70.4
Urge the ED to make arrangements so that nurses can get medical care as needed for both themselves and their families.	37	19.9	53	28.5	96	51.6
Watch and alert medical supply members to supply shortages	36	19.4	48	25.8	102	54.8
Have a strategy for emergencies that includes job requirements and potential substitute responsibilities and locations for at-risk staff (such as pregnant employees and other designated risk categories).	19	10.2	51	27.4	116	62.4
Prepare guidelines for conservative and re-use of N95 respirators/powered air-purifying respirators (PAPR) if severe shortages are coming up	17	9.1	70	37.6	99	53.2
Create a hospital pandemic safety plan, and designate a safety officer to make any necessary modifications.	41	22	32	17.2	113	60.8
Evaluate the need for family support to enable nurses to work (e.g., childcare)	14	7.5	27	14.5	145	78
Provide information for family care plans that are designed to guide caregivers through providing the important details about childcare, school, medical care, and family activities	14	7.5	33	17.7	139	74.7
Create a unit (ED) pandemic safety strategy and designate a safety officer to make any necessary modifications.	13	7	49	26.3	124	66.7

The most crucial educational subjects for preparing ER nurses to care for pediatric patients who are critically sick with infectious diseases were ranked as the notion of crisis standards of care (34.9%) and creating an emergency plan (plan B) in case of a supply shortage (30.6%). To effectively care for pediatric patients who are critically ill with communicable diseases, other highly ranked topics included developing palliative care plans for outbreak victims and their families (23.1%), patient assessment priority (21.5%), and communicable illness screening procedure (20.4%). However, according to nurses, safety and infection control during communicable disease epidemics, proactive planning in which leaders plan for worst-case scenarios—the development of patient information sheets, care plans for communicable disease epidemics, and communication pathways (19.4%, 13.4%, 9.7%, and 5.4%, respectively) were the least important educational topics (Table 3).

**Table 3:** Ranking of the pandemic educational demands according to importance (N = 186).

Communicable disease pandemic educational topics	Frequency	Percentage
The principles of Crisis Standards of Care (CSC)	65	34.9
How to prepare an emergency plan (plan B) in case of shortage in supplies.	57	30.6
Develop palliative care plans for communicable disease epidemics patients and their families.	43	23.1
Patient assessment and reassessment priorities.	40	21.5
The screening process of communicable disease epidemics	38	20.4
Safety / Infection Control of communicable disease epidemics.	36	19.4
Proactive planning, in which leaders anticipate and take steps to address worst-case scenarios, is the first link in the chain to reducing morbidity, mortality, and other undesirable effects of an emerging disaster.	25	13.4
Develop care plans for communicable disease epidemics.	18	9.7
Develop /provide patient information sheets, and communication pathway.	10	5.4

## Discussion

The purpose of this study was to assess the nurses’ readiness to provide care for pediatric patients with infectious diseases. Managing the enormous influx of at-risk pediatric patients during infectious disease outbreaks may be challenging for nurses who choose to work in emergency rooms [17]. Are nurses also competent in handling pediatric infectious illness emergencies? [18,19]. It’s possible that they didn’t have enough training to supervise the infection control preventative procedures. How the evidence-based practice paradigm might be enhanced in the future to better manage infection in pediatric patients undergoing emergency care? Also, for community safety, activities for potential emergency infectious diseases need to be prepared for [18].

It may be possible to increase patient safety and pediatric patient prognosis by understanding the current state of hospital preparation for pediatric infectious disease emergencies. Patient safety can be achieved via proactive continuous risk reduction, ongoing assistance with effective responses to real accidents, and other methods [6,20–22]. Identifying potential risks and hazards as well as putting policies in place to lessen the possibility of an infectious disease epidemic are part of this. For instance, hospitals can put in place infection control procedures like hand hygiene guidelines, environmental cleaning, and isolation precautions to stop the spread of dangerous diseases.

Further, to proactively reducing risk, hospitals should be prepared to respond to infectious disease emergencies when they occur [18]. In hospitals, the planning process could be challenging. In order to organize an activity, this necessitates having trained individuals, such as nurses, appropriate equipment and materials, and open lines of communication. Nursing professionals also need to be aware of the special requirements of pediatric patients, such as the proper administration of drugs, keeping an eye out for side effects, and offering both the patient and their family emotional support [19].

Participants reported they had received inadequate training in pediatric infectious illness emergency planning methods. The results are in line with the Chanie et al. (2021) study, in which nurses and other healthcare professionals acknowledged being underprepared for infectious disease situations [23]. This finding could be explained by a variety of variables, including informal training in infectious disease emergencies (i.e., using both personal and professional experiences) and a significant amount of trial-and-error learning when learning how to treat high-risk patients, especially pediatric patients [24]. Likewise, inadequate hands-on training had a detrimental impact on the nurses’ ability to provide appropriate and safe care for patients who pose a risk [25]. Combined, these findings examine the necessity of consistent and ongoing training for hospital and unit-based pandemic preparation programs [11], especially for nurses with age-specific infection prevention and control competencies for pediatric patients.

Moreover, participants reported that "evaluating the need for family assistance to enable nurses to work" and "providing specifics for family care plans that are intended to help caregivers by instructing them on how to supply the crucial information concerning childcare, school, medical care, and family activities" were the infection prevention and control tasks that, when dealing with an emergency of infectious disease, had the worst performance. This finding could be explained by the fact that nurses are more likely to struggle with issues and worry about spreading illnesses to their family members because they might have elderly relatives or young children living in their home [26].

Furthermore, participants stated that developing an emergency plan should focus on evaluating the present level of training requirements, the amount to which routine precautions are taken, the equipment’s availability and suitability, and what the plan is in the event of a serious shortage. The finding is in line with the findings of the Al Haliq et al. (2023) study, which found that the training and education of infectious disease crisis preparedness were insufficient with regards, the development of infectious disease crisis preparedness plan [6].

More, participants reported that the operation of the infectious disease emergency safety plan at the unit and hospital level with a designated expert in safety and determining an emergency plan with job requirements and suitable replacement responsibilities and locations for at-risk staff (such as pregnant employees and other designated risk categories) was subpar. The finding is in line with the findings of the Al Haliq et al. (2023) study [6]. This is indicated by OSHA’s recommendation (2020) to apply the "hierarchy of controls" approach when evaluating approaches to reduce workplace risks. Effective controls don’t rely on employee behavior; instead, they eliminate the risk. Examples include developing a safety plan with a designated safety expert at the unit and hospital levels and coming up with an emergency plan for workers who are at danger [27,28].

Participants also reported that the Inventory control procedure didn’t work well. The outcomes are in line with those of [6,29]. This can be attributed to hospitals not having a tracking system that would enable them to keep track of approaching acute shortages and alert the unit and hospital earlier. As well, participants agreed that a system must be created to make it simpler for nurses and their families to access medical care and to brush up on their infection prevention skills. This emphasizes how essential it is for emergency departments to be prepared for a possible pandemic. In order to respond to any emergency efficiently, safely, and with equity at the forefront, also, to protect the mental health and wellness of nurses working in the emergency department, a modernized response system must be constructed.

Besides, the notion of crisis standards of care, developing an emergency plan (plan B) in case of a supply shortage, developing palliative care plans for outbreak victims and their families, patient assessment priority, communicable disease screening procedure, and clarification of communication pathways were ranked as the relative importance of the pandemic’s educational demands. The Crisis Standards of Care (CSC) framework aids healthcare professionals in making decisions during public health emergencies when resources are limited and demand exceeds supply. This approach is crucial for pediatric nursing emergencies during pandemics where there is a high danger of infection transmission and where children’s demands may differ from those of adults [30]. Prioritizing children’s needs, distributing resources fairly, preserving effective communication, ensuring continuity of care, preparing for staffing shortages, offering education and training, and continuously assessing and improving the response to the pandemic are all part of the CSC of pandemic infection control of pediatric nursing emergency principles.

A crucial component of emergency preparedness model is creating a backup plan (Plan B) in case of supply shortages. It can be made by listing the supplies that are vital to your operations and the care of your patients, including medicines, medical equipment, personal protection equipment, and other necessary goods. Then, categorize the items on a list according to priority and the possibility of shortages, and create backup plans that identify alternate sources of supply like other manufacturers or suppliers. It is critical to establish clear communication lines with suppliers, healthcare professionals, and other stakeholders to ensure awareness of any. Additionally, nurses need to be taught the emergency plan and what to do in case of a shortage. This can entail following protocols for restricting supplies, employing substitute supplies, or putting infection control measures into place. To ensure that the strategy remains current and effective in addressing any possible shortages, monitor, assess, and update it frequently. These procedures can help nurses create a thorough emergency plan (Plan B) to overcome supply shortages in an emergency. Prioritizing patient care while protecting nurse provider safety, being flexible to changing circumstances, and prioritizing patient care are all important aspects of the action plan [7]. On top, enhancing the quality of life for patients and their families who are struggling with serious illnesses is another goal of palliative care. To manage their symptoms and provide comfort, pediatric patients who contract an infectious disease during a pandemic may require palliative care [31].

This strategy calls for an all-encompassing strategy that addresses the patient’s and family’s needs, treats symptoms, and offers psychological and spiritual support. To guarantee that the patient receives the best care possible, coordination and continuity of care are crucial [31]. Finally, nursing assessment and reassessment should place a high priority on stabilizing the Airway, Breathing, and Circulation (ABC) before assessing symptoms, gathering medical and exposure history, determining mental status, managing pain, offering emotional and psychosocial support [26], and frequent reassessment when caring for pediatric patients with communicable diseases in the Emergency Room (ER) [21,32].

## Limitations

Our findings have numerous limitations. First, we used a convenience sample, so the participants who completed the survey may only fully reflect the readiness of those who did not. This may restrict the study’s generalizability. Second, the sample size was limited to three tertiary hospitals in Amman, Jordan’s capital; each hospital has different resources and capabilities, limiting the external validity of the findings. Lastly, using a self-report questionnaire may introduce bias because participants may not always precisely describe their pediatric experience with communicable disease.

## Conclusions

The main aim of this study was to assess the emergency nurses’ readiness to provide care for pediatric patients with infectious diseases. According to the findings, there was insufficient training in infectious disease emergency prevention and control for pediatric patients. As evidenced by the low percentage of participants who reported having received training. As a result, nurses and healthcare systems are strongly urged to participate in structured training programs on a regular basis to strengthen their preparedness for any infectious disease [33].

In addition, this study displays that the least-implemented procedures were family support plan, a backup plan that includes (standard precautions, training requirements, and equipment), unit and hospital pandemic safety plan, strategic emergency plan for at-risk staff such as (pregnant employees and other designated risk categories), inventory control plan, a system that will make it easier for nurses and their families to seek medical treatment, and create a nurse return-to-work policy for those who become ill.

It is highly recommended for nursing education programs to include modules on specific pediatric infectious diseases by offering specialized courses or modules that address pediatric infectious illnesses that are commonly seen in emergency rooms [1]. Also, ensure that nursing education includes thorough teaching of hand hygiene, the use of personal protective equipment (PPE), isolation precautions, and suitable disinfection and sterilization techniques [13].

Furthermore, this study highlights simulation-based training to improve nursing abilities and decision-making when managing viral infections in pediatric patients. Ensure that nurses can access credible, fact-based information about pediatric infectious diseases. Arrange clinical rotations at pediatric infectious disease departments or emergency rooms. During these rotations, nurses can receive practical experience treating children and patients with infectious disorders. This conclusion was also supported by another study [1].

Thus, Jordan’s nursing quality of care will be affected in the future due to a lack of information regarding caring for children’s patients with infectious disorders. A study in this field can focus on a variety of topics, including investigating the prevalence, incidence, and transmission patterns of infectious diseases in children’s populations, which may aid in determining risk factors and developing effective defence mechanisms.

More research should be conducted to improve diagnostic procedures for the accurate and timely detection of infectious illnesses in children. Analysing the outcomes of public health efforts such as school policies, community-based interventions, and vaccination campaigns can provide insight into how effectively they perform to prevent and control communicable diseases in children.

## Supporting information

S1 Dataset (XLSX)
